RETRACTED

# Metagenomics for taxonomy profiling: tools and approaches

**DOI:** 10.1080/21655979.2020.1736238

**Published:** 2020-03-09

**Authors:** Mukesh Kumar Awasthi, B. Ravindran, Surendra Sarsaiya, Hongyu Chen, Steven Wainaina, Ekta Singh, Tao Liu, Sunil Kumar, Ashok Pandey, Lal Singh, Zengqiang Zhang

**Affiliations:** a College of Natural Resources and Environment, Northwest A&F University, Yangling, Shaanxi Province, China; b Swedish Centre for Resource Recovery, University of Borås, Borås, Sweden; c Department of Environmental Energy and Engineering, Kyonggi University Youngtong-Gu, Suwon, South Korea; d Key Laboratory of Basic Pharmacology of Ministry of Education, Zunyi Medical University, Zunyi, Guizhou, China; e Institute of Biology, Freie Universität Berlin Altensteinstr, Berlin, Germany; f CSIR-National Environmental Engineering Research Institute, Nagpur, India; g Centre for Innovation and Translational Research CSIR-Indian Institute of Toxicology Research, Lucknow, India

**Keywords:** metagenomics, genomics, deoxyribonucleic acid, ribose nucleic acid, microbial metagenomes

## Abstract

The study of metagenomics is an emerging field that identifies the total genetic materials in an organism along with the set of all genetic materials like deoxyribonucleic acid and ribose nucleic acid, which play a key role with the maintenance of cellular functions. The best part of this technology is that it gives more flexibility to environmental microbiologists to instantly pioneer the immense genetic variability of microbial communities. However, it is intensively complex to identify the suitable sequencing measures of any specific gene that can exclusively indicate the involvement of microbial metagenomes and be able to advance valuable results about these communities. This review provides an overview of the metagenomic advancement that has been advantageous for aggregation of more knowledge about speciﬁc genes, microbial communities and its metabolic pathways. More speciﬁc drawbacks of metagenomes technology mainly depend on sequence-based analysis. Therefore, this ‘targeted based metagenomics’ approach will give comprehensive knowledge about the ecological, evolutionary and functional sequence of significantly important genes that naturally exist in living beings either human, animal and microorganisms from distinctive ecosystems.

## 1. Introduction

Since the invention of the microscope and other analogous observational instruments that could be exploited to explore the micro world, we humans are becoming conscious that microorganisms are of equal significance with plants and animals and have played a vital role in the dynamic derivation of earth bio geosphere. With the passage of time, scientists recognized that a single study of one pure species in the laboratory scale contradicts laws of nature, since organisms cannot survive and grow as one single species. They could only exist as a member of interdependent communities in various natural environments. Thus, the amount of microbes existing in nature cannot be incubated alone in the laboratory. Hence, in order to establish gene inventories, a further better understanding to functions of populations and communities in an ecosystem, etc., is necessary and inevitable to study the hereditary information of all entangled species. In 1998, ‘metagenomic’ was first proposed as ‘the collective genomes of soil microflora’ and approached to investigate genetic information of all populations [1]. Later, ‘metagenomic’ was defined as ‘the functional and sequence-based analysis of the collective microbial genomes that are contained in an environmental sample’ by Allen and Banfield [2] and Cowan et al. [3]. Since the first application of metagenomics, now it has been comprehensively utilized to study microbial diversities in a certain environmental community by analyzing selected genes such as 16 S rRNA.

RETRACTED

### 1.1. Classification of metagenomic

The purpose of the taxonomic classification of metagenomic sequences is to find the exact species of origin, data of which are also primarily performed with the objective of cataloging/classifying various microbial groups inhabiting a given environment. Therefore, taxonomic classification is a crucial procedure for different applications of metagenomic such as disease diagnostics, microbiome analyses, and outbreak tracing, etc. Current taxonomic classification algorithms mainly utilize handcrafted sequence composition features such as oligonucleotide frequency [4,5].

Given massive bio-sequencing data, it is extremely critical to efficiently analyze the categories of these biological sequences within a limited time, so as to capture characteristics of the microbial community which researchers are interested in. Afterward, researchers can further investigate the species diversity of microbial communities by applying classification methods of metagenomics samples to classify sequencing data from environmental samples. The metagenomics sample classification methods study the relationship between changes of environmental or host state and microbial community by identifying or predicting categories of metagenomics samples. The classification methods of metagenomics sequencing data can be divided into two categories according to different sample data processed methods: one is based on the sequence of marker genes such as 16SrRNA, the other is based on whole-genome sequencing fragments.

RETRACTED

### 1.2. Basic tools and techniques used in metagenomic

Metagenomic is based on genetic recombinant technology. The general procedure for metagenomic research has been depicted in Figure 1, which generally includes the enrichment of samples or genes (groups), extraction of genomic DNA in a specific environment, construction of metagenomic DNA library, screening of the target gene, and expression of active product of the target gene. Among them, the methods of direct cracking and indirect extraction are two conventional technologies used for DNA enrichment and extraction from environmental samples in the metagenomic analysis. DNA from the samples should be extracted completely and maintain larger fragments to obtain unbroken target genes or gene clusters as much as possible. The construction of the genomic library is a prerequisite for revealing new genes. During this procedure, the choice of vector and host system depends on the quality of extracted DNA and purpose of research, which the size of insert, number of vector copies required, host selected as well as screening methods all need to be taken into consideration. The next step is to effectively utilize the abundant resources of the library to discover new biomolecules. Due to the high complexity of the environmental genome, high-throughput and highly sensitive technologies are required to screen and identify useful genes in libraries. Currently, widely adopted screening technologies can be broadly divided into four categories: function-driven screening, sequence-driven screening, SIGEX (substrate-induced gene-expression) screening and compound configuration screening.

With the expeditious development of the metagenomic research in recent years, the quantity of sequencing microbial genomes increased exponentially, which means that the comparison requirement for novel sequencing reads is also synchronously increasing. This requests the development of efficient tools which could analysis metagenomics data accurately. Numerous tools have been exploited to classify metagenomic data and estimate taxon abundance profiles. Table 1 compares the characteristics of various classifiers that are commonly chosen to apply in metagenomics technologies.

**Table 1.** Characteristics of different classifiers.

Type	Classifier	Custom databases	Generates abundance profile	Memory required	Time required	Reference
DNA	CLARK	Yes	Yes	80 Gb	2 min	[119]
	Kraken	Yes	Yes	190 Gb	1 min	[120]
	MegaBLAST	Yes	No	61 Gb	4 h	[121]
	Prophyle	Yes	No	40 Gb	40 min	[122]
Protein	DIAMOND	Yes	No	110 Gb (varies)	10 min	[123]
Markers	MetaPhlAn2	No	Yes	2 Gb	1 min	[124]
	mOTUs2	No	Yes	2 Gb	1 min	[125]

RETRACTED

**Table 2.** Correlation between soil physicochemical parameters and bacterial OTUs.

Taxa	Parameters	Positive correlation (+) and negative correlation (-)	References
Proteobacteria	pH	+	[126]
	Total organic carbon	+	[127]
	Total nitrogen	+	[128]
	Phosphorus	+	[129]
Actinobacteria	pH	+	[130]
	Total organic carbon	-	[126]
	Total nitrogen	-	[126]
	Phosphorus	-	[126]
Acidobacteria	pH	-	[128]
	Total organic carbon	+	[124]
	Total nitrogen	+	[125]
	Phosphorus	+	[127]
Firmicutes	pH	-	[129]
	Total organic carbon	+	[124]
	Total nitrogen	ns	[125]
	Phosphorus	ns	[128]
Bacteroidetes	pH	+	[123]
	Total organic carbon	-	[124]
	Total nitrogen	-	[125]
	Phosphorus	+	[125]
Verrucomicrobia	pH	-	[121]
	Total organic carbon	+	[124]
	Total nitrogen	ns	[130]
	Phosphorus	+	[130]
Planctomycetes	pH	-	[131]
	Total organic carbon	+	[121]
	Total nitrogen	+	[125]
	Phosphorus	+	[125]
Cyanobacteria	pH	-	[132]
	Total organic carbon	+	[132]
	Total nitrogen	+	[133]
	Phosphorus	ns	[125]
Armatimonadetes	pH	+	[125]
	Total organic carbon	-	[125]
	Total nitrogen	-	[125]
	Phosphorus	ns	[125]
Chloroflexi	pH	+	[134]
	Total organic carbon	ns	[125]
	Total nitrogen	-	[125]
	Phosphorus	ns	[135]

ns – no significance.

**Table 3.** Summary of recent research literature on the microbial community.

Region	Year	Published research themes	Process, tools and techniques	Key research outcomes	References
Saudi Arabia	2020	Metagenomics-based evaluation of microbial profiles	Shotgun metagenomic tools; CosmosID metagenomic software; high performance k-mer algorithm databases	Metagenomics revealed a lower alpha diversity for both bacteria and virus	[85]
United States of America	2019	Whole metagenomic sequencing for microbial community	Whole metagenome sequencing; Descriptive analyses using SAS® 9.4	whole metagenomics approach to characterize sediment microbial biodiversity	[63]
China	2019	Metagenomic sequencing for microbial gene catalog	Metagenomic sequencing using an Illumina Hiseq 2000 sequencing system; MetaGene predicted an open reading frames (ORFs); Gene taxonomic classification using BLASTP search	Metagenomic sequencing is conducted to investigate the microbial gene catalog	[62]
Singapore	2019	Bioinformatics analysis of metagenomics data of biogas-producing microbial communities	Next-generation sequencing (NGS) technologies used for qualitative and quantitative analysis of the microbial communities	Described the procedure of processing metagenomics data of microbial communities for revealing metagenomics characterization using bioinformatics approaches	[86]
China	2019	Metatranscriptomics for rhizosphere microbiomes	Random-primed cDNA libraries using the NEBNext Ultra Directional RNA Library Prep Kit for Illumina; The cDNA libraries using the Experion DNA 12 K Analysis Kit (Bio-Rad) and quantified using the Qubit dsDNA HS Assay kit	Metatranscriptomics revealed significant eCO2 effects on the composition and activity of the grassland microbiomes	[87]
China	2020	Metagenomic insights for microbial community and antimicrobial resistance genes	Shotgun metagenomics sequences processed using Trimmomatic 0.36 and Bowtie2 via the KneadData wrapper software; MEGAHIT v1.1.3 used for de novo metagenomic assembly analyses; The draft genomes annotated using Prokka software and eggNOG-mapper (based on eggNOG 4.5 orthology	The results give first metagenomic insights into the salt-mediated changes in microbial community composition and a broad view of associated antibiotic resistance genes in the process of food fermentation.	[134]
Canada	2018	Mining metagenomic and metatranscriptomic data for microbial metabolic functions	Metagenomics and metatranscriptomics, including nucleic acid extraction, sequencing platform selection, library construction, quality control of sequencing outputs, compositional analysis, assembly-based functional analysis, assembly-free functional analysis, and comparative analysis.	Metagenomics and metatranscriptomics can arrest the whole genome and transcriptome range of microorganisms through sequencing entire DNA/RNA, providing both taxonomic and functional information with high resolution	[69]
Switzerland and Israel		Microbial Metagenomics Mock Scenario-based Sample Simulation (M3S3)	Microbial Metagenomics Mock Scenario-based Sample Simulation (M3S3) workflow generate virtual samples from raw reads or assemblies	The M3S3 tool is support the progress and authentication of identical metagenomics applications	[88]

RETRACTED

## 2. Novel biological resources screened from uncultured bacteria by metagenomic method

Nowadays, more than 99% of microorganisms are currently difficult or cannot be purely cultured in microbiology field, which means our knowledge of microbes is basically limited in less than 1% of microorganisms [1]. Those uncultured microorganisms possess great application potential, their metabolites may produce amounts of valuable compounds. The emergence and development of metagenomic have made up for this deficiency and serve us commence to gradually explore and understand the potential micro-world. It has been widely recognized that metagenomic can be utilized to discover novel genes, enzymes, as well as compounds from uncultured bacteria. Currently, researchers have employed metagenomic to obtain numerous novel functional genes and active substances, which have been extensively applied in various fields. Two primary categories are ordinarily utilized in metagenomic to discover and identify novel natural genes and compounds from environmental samples, which are sequence-based screening and function-based screening, respectively. For sequence-based screening, the PCR technology is employed to detect the existence of genes and compounds, while function-based screening in metagenomic is conducted by investigating the activity of enzymes [6–8]. These two technologies have deciphered amounts of novel genes encoding valuable biocatalysts from uncultured bacteria existing in different specific environments, which have already been broadly practiced in many industries such as environmental restoration, new medical compounds, and alternative energy, etc.

RETRACTED

In addition, notable companies include DNA Star, Inc (US), Illumina, Inc. (US), Oxford Nanopore Technologies Ltd. (UK), IntegraGen SA (France), Macrogen Inc. (South Korea), Thermo Fisher Scientific, Inc (US), Novogene Corporation (China), Allwegene Co. Ltd (China), CD Genomics (USA), BGI (USA), Zymo Research Corporation (US) and Microsynth AG (Switzerland) that are providing services regarding metagenomic analysis.

## 3. Metagenomic analysis and its applications in different sector

### 3.1. Agriculture

In the last few decades, the production of crops has been increased worldwide. The quality of soil can alter plant production in agricultural soil. In general, the soil system contains an enormous amount of microbial population (e.g., 10 billion microbes/gram) as well documented by Rosselló-Mora and Amann [9]. Microorganisms and their metabolic activities can enhance crop production [10,11]. In addition, agriculture is playing an important role in the world economy [11,12]. Therefore, there is an urgent requirement of metagenomic analyses to understand the microbial communities in the soil system [13]. The metagenomic analysis is normally used to examine various microbial communities from the environment (Figure 4). The microbes can stimulate the cycling of macro as well as micronutrients and also microbes release the essential enzymes which enhance crop production [14]. Metabolic network and modeling of microorganisms provide the information on various biochemical activities [13]. At present, an enormous number of metabolic re-constructions associated with microorganisms have been modeled [15,16]. Metabolic rebuild of microorganisms, namely, *Saccharomyces cerevisiae* and *Escherichia coli* is analyzed using the dynamic flux balance analysis [17]. According to previous literature, metagenomic models were not well addressed. These approaches can detect the metabolic features from sequence data.

### 3.2. Biofuel

Due to the growing interest of minimizing the negative environmental impacts accompanied by the utilization of petroleum during energy production, alternative energy sources, such as biofuels, are being explored [18]. The availability of feedstocks needed for the production of biofuels (e.g. waste gas, biomass and organic residues) can be largely guaranteed [18–20]. The types of biofuels that can be produced include bioethanol, biogas, biohydrogen, and biodiesel [18,21]. The bioconversion of the waste materials and residues into biofuels involves biochemical reactions that essentially control the microbial activities [22]. During the bioconversion process, metagenomic analysis is critical in characterizing the functional microbial communities involved as well as the associated metabolic pathways [23]. The metagenomic analysis tools can also be applied during the biologically mediated substrate preparation steps prior to the actual fermentation. For instance, Kundu et al. [24] classified the metabolic interaction network of gut compartments of *Nasutitermes corniger* used for lignin disintegration. The pretreatment of lignin-rich materials is critical for biomass utilization in the bioethanol production process [25]. Biogas is produced when organic materials are broken down in oxygen-deficient conditions in the so-called anaerobic digestion process catalyzed by naturally-occurring microflora. The process involves four interdependent stages facilitated by hydrolytic, acidogenic, acetogenic, and methanogenic microbes (Table 2). The diverse groups of microorganisms that are active during the biogas production process have been studied by several authors [18,23,26].

RETRACTED

A remarkable research that was conducted by Campanaro et al. [27] revealed the phylogenetic and functional structure of the microbial population in bioreactors digesting cattle manure. Their novel approach entailed the application of high-throughput sequencing and binning procedures which resulted in a comprehensive report on the metabolic pathways involved. Biohydrogen can be produced in anaerobic digesters in the acidogenic and acetogenic steps, alongside other metabolites such as volatile fatty acids (VFAs) [28]. When the anaerobic digestion processes are aimed at these intermediate metabolites, the activity of methanogenic archaea must be deactivated while appropriate methods are applied to manipulate the microbial pathways toward the targeted product [29]. The VFAs are potential precursors in the biodiesel production process due to their use as carbon sources for cultivating oleaginous microbes [30]. The identification of bacteria responsible for the acidogenic fermentation has been widely performed, sometimes alongside the methanogenic archaea profiling [27,31,32]. Some of the analytical tools that can be mentioned include 454 pyrosequencing and fluorescent in situ hybridization (FISH) [33].

RETRACTED

Microalgae are promising microorganisms that can also be used to synthesize biofuels coupled with CO_2_ fixation [34]. Metagenomic analysis has also been performed on these microorganisms. For instance, Sambles et al. [35] used high-throughput Illumina sequencing and 16S rDNA analysis to study the microbial composition of *Botryococcus braunii* at diverse treatments. The microbial analysis is also crucial in understanding other important components during the bioprocessing of microalgae, such as biofouling of photo-bioreactors [36]. A previous research was conducted to identify the metagenome of a bacterial biofilm in a photo-bioreactor using 16S rRNA phylogeny after which a KEGG pathway analysis was performed. The bacterial species originated from *Chlorella vulgaris* and *Scenedesmus obliquus* [36].

### 3.3. Biotechnology

In the present century, various molecular techniques include terminal restriction fragment length polymorphism (T-RFLP), denaturing gradient gel electrophoresis (DGGE), polymerase chain reaction (PCR) cloning, fluorescence in situ hybridization (FISH) are applied to microorganisms, these modified microbes contain different applications [37–39]. These microbial techniques can enhance the knowledge in the field of microbiology, but the interaction of microbes and their mechanisms are not well addressed. Metagenomics is one of the suitable methods to study microbial genetics collected from various environmental samples [40]. Furthermore, metagenomics has provided the whole-genome sequences of microorganisms [41–43]. Metagenomics is also used and examined the metatranscriptomes from recovered samples to detect the microbes and their gene expression [44,45]. Moreover, many scientists have been using metagenomics to detect the novel microbial genes for biodegradation and also monitoring the biohazards associated with microorganisms (*i.e*., viruses, various pathogens and, ARGs) as well documented by Wexler et al. [41] and Xia et al. [46].

### 3.4. Ecology

The ecosystem contains many types of microorganisms which regulate the different biological processes and biogeochemical cycles. The large level of microbial diversity can enhance ecosystem stability and productivity [47–49]. Understanding of microbe’s interaction between living organisms and their internal mechanisms from the molecular view. Metagenomic methods are promising tools for analyses of microbial ecosystems [50–52].

### 3.5. Environmental remediation

The major sources of environmental pollution associated with industrial based on wastewater/wastewater sludge. In general, industries are consumed different types of chemical substances for the production of various materials and release several hazardous substances at the end of the process. Various industries release different types of hazardous waste materials (e.g., polyaromatic hydrocarbons, phenols, pesticides and toxic heavy metals) which generate serious environmental pollution [53–56]. Bioremediation is environment-friendly and low-cost technology to the reclamation of polluted soils, particularly microbes play an important role in biodegradation of pollutants [53,55,57,58]. Active microbes in contaminated sites can be assessed by genome enhancement using metagenomic analysis (Figure 2). Particularly, stable isotope probing (SIP) techniques employing for enhancement of different macromolecules include RNA, DNA, phospholipid-derived fatty acids [59]. Metagenomic methods are one of the emerging techniques for sequences of various microbes and enhanced microbes through metagenomics can remove the different pollutants from the contaminated environment.

RETRACTED

### 3.6. Pharmaceutical and medical science

At present, many more peoples are affected by various diseases particularly type 1 diabetes, bowel disease (IBD), Crohn’s disease and ulcerative colitis. These diseases severely affected the human immune system. In addition, weakness alleles have generated deadly diseases in human beings. Apart from this, some microorganisms can contribute to pathogenesis. The detection of proteins associated with pathogenesis is very complicated. Metagenomics-based technologies can identify specific genes [60,61].

## 4. Microbial metagenomics, metatranscriptomics, and metaproteomics

### 4.1. Microbial metagenomics

With the rapid advancement of high-throughput sequencing, a cultivation-independent methodology, i.e., metagenomics, can become a competent approach to the examination of the ability of certain microbes for refining. Metagenomic microbial sequencing is a competent alternative to rRNA sequencing to examine the complex microbial community structure, and allow screening of a microbial community’s innate composition and utilitarian potential [62]. The development of sophisticated molecular approaches in conjunction with computational regulations has resulted in a decline in the sequencing of aggregate genome DNA and several opportunities related to marine microbial exploration (Figure 5). As a result, an entire era of metagenomic sequencing has contributed to more in-depth considerations of representing a wider range of species from varying tests [63–66]. Li et al. [67] showed that metagenomics-based population analyses can provide both community and valuable information without an upgrade slant. This approach has been utilized for comparing functional and requested profiles of the microbial communities related to specific types.

RETRACTED

Commercial devices have risen which are arranged to address this issue by upgrading for microbial DNA. One methodology, Unused Britain Biolab’s NEB Next Microbiome DNA Improvement unit, takes advantage of human and other higher orchestrate eukaryotic DNA having tall CpG methylation rates. By utilizing the methylated CpG-specific official protein MBD2 entwined to a human IgG Fc portion, human DNA is particularly bound and confined utilizing Protein A-bound attractive dots [68]. Multiple omics methods are used to govern the microbial community alignment, co-occurrence network along with metabolic pathways. Deng et al. [69] hypothesis revealed that niche transformations caused a distinct microbial assembly and increased microbial ecology circulation, which has the possibility to improve system effectiveness and stability. The higher microbial diversity, efficient redundancy and observed higher system stability are related to the huge niche differences in reactors [69]. Deng et al. [70] research further revealed a similar difference trend in the phylum taxonomy level between floc bacteria and gut microbiota. The microbial community distribution for both water and gut samples was visualized by principal coordinate analysis (PCoA) based on the detected operational taxonomic unit.

### 4.2. Metatranscriptomics

Metagenomics and metatranscriptomics can collect the microorganism’s entire genome and transcriptome range by sequencing add up to DNA/RNA from different natural tests, delivering useful data with high determination. The metatranscriptomics represents valuable devices for all-inclusive cataloging microbial quality and transcript profiles and reflecting generally metabolic capacities [71]. Falk et al. [72] uncovered that microbial genomic potential can be remade by metagenomic investigation of environmentally extracted DNA, metatranscriptomics can shed light on the deciphered items of DNA, giving riches of data on add up to flag-bearer RNA (mRNA) yield; an intermediary for quality expression. As microorganisms are coupled to numerous biogeochemical cycles within the environment, metatranscriptomic considers of anthropogenically affected dregs are profitable in numerous aspects; 1) understanding critical reactions of the biosphere to irritations, 2) evaluating in case and how microbial communities are working to direct the impacts of bequest defilement in oceanic frameworks, and 3) investigating microbial differing qualities as a work of human-induced scene changes. As of late, metagenomic or metatranscriptomic examinations of Italian cheese, French cheese, Mexican cheese and Belgian cheese have been performed, creating modern information with respect to differences and metabolic highlights of microbial species in cheeses [73].

RETRACTED

With the improvement of microarray and high-throughput sequencing, the metatranscriptomics has uncovered the startling high microbial differences in corrosive mine seepage, which given a profound knowledge that a much larger assortment of life forms may adjust to this extraordinary environment than already thought. Genome and transcriptome investigations had given an expansive sum of quality data about potential capacities of acidophiles, particularly within the metabolic pathways of carbon, nitrogen, hydrogen and sulfur Liyuan et al. [74]. Lim et al. [75] uncovered that metatranscriptomics of host-associated communities is especially troublesome. Enhancement of the microbial RNA by strategies that utilize manufactured polyadenylation is not pertinent for tests that contain huge amounts of eukaryotic mRNA. The added poly-A tails decrease the sum of valuable arrangement information, particularly when pyrosequencing advances such as Roche/454 are utilized. Due to the brief half-life and small amount of mRNA, test filtration and control with buffer ought to be dodged earlier to RNA extraction. This definitely causes an increment in host RNA defilement when managing with host-associated microbial tests. Metatranscriptomics uncovered critical eCO_2_ impacts on the composition and movement of the meadow microbiomes. The decrease in soil parasitic movement was affirmed by RT-qPCR of 18S rRNA; in great agreement with a noteworthy diminish in contagious mRNA included in oxidative phosphorylation (rhizosphere soil), and in collapsing, sorting and debasement (root-associated). Among Organisms, the relative plenitude of most bunches (e.g., *Agaricomycetes* [soil] and *Leotiomycetes* [roots]) diminished, but that of the *Glomeromycetes* (both compartments) expanded. Utilitarian investigation of root mRNA recommends that the generation of plant auxiliary metabolites was expanded within the summer [76]. Besides, the effect of worldwide warming on the endophytic and epiphytic living beings related with *C. quitensis* remains unclear. Here, a metatranscriptomic approach was utilized to decide the impact of an in situ reenacted worldwide warming situation on *C. quitensis* plants. We found a huge number of differentially communicated qualities effectively explained (2997), recommending that climate alter tweaks the metatranscriptome of *C. quitensis* plants and related endophytes and epiphytes [77–79].

RETRACTED

### 4.3. Metaproteomics

Recently, metaproteomics and metabolomics have emerged as effective devices for the characterization of energetic host–microbiome interactions, especially in combination with metagenomics and metatranscriptomics approaches [80]. Metaproteomics can be utilized to consider protein expression from blended cultures and thus this approach can supply coordinate to prove the metabolic and physiological exercises occurring in a given framework (Figure 3). This approach has been utilized somewhere else to consider the relationship between the structure of microbial communities and the working of a biological system [81]. Soil metaproteomics has the potential to contribute to be distant for a better higher understanding of warming impacts on soil living beings as proteins especially talk to dynamic living beings and their physiological working. The contrasts in community work may be related to particular phyla utilizing metaproteomics, showing that microbial adjustment to long-term soil warming basically changed microbial capacities, which is related to upgraded soil breath [82]. Metaproteomics exploits the control of mass spectrometry to recognize wide protein profiles in complex tests, such as digestive tract microbiota. The foremost recent mechanical advances inside the field of mass spectrometry have opened the field of large-scale characterization of microbial proteins. In spite of these hardware progressions, bioinformatics examination remains a fundamental challenge [83].

Shotgun metaproteomics may uncover the functional geography of microbial population, but needs suitable strategies for complicated tests with obscure formulations. Beyter et al. [84] have displayed Proteo-Storm, a competitive database looks like a framework for large-scale metaproteomics that identifies high-confidence peptide-spectrum matches while accomplishing a speedup of two-to-three orders-of-magnitude over reigning systems. Metaproteomics could be an effective tool for getting information on all proteins recuperated specifically from natural tests at a given time. The proteome information gives to coordinate prove on the biological processes in the soil environment and is the primary detailed reference information from the maize rhizosphere(Table 3). The LC-MS/MS proteomic information is accessible by ProteomeXchange with identifier PXD014519 [85]. The induction of proteins from the respective peptides and the confirmation of the source and function of these proteins are the major steps toward meta-proteomics information analysis. In this way, the instructional exercise introduces the Unipept command-line interface as a platform-independent method for such metaproteomics knowledge assessments. To continue with, the open Unipept commands are given point by point. Next is the regulation of the Unipept command-line interface utilizing two case studies examining a single tryptic peptide and a group of peptides retrieved independently of a shotgun metagenomics test [86].

RETRACTED

## 5. Metagenome analysis and interpretation

Metagenomics uncovered a lower alpha difference for microbes from different sources. The current approaches to recognizing changes in the microbial community incorporate qualitative approaches like terminal restriction fragment length polymorphism (T-RFLP) or quantitative approaches like real-time PCR (qPCR). T-RFLP produces fingerprinting profiles for comparative investigation but does not give data on the ordered personalities of microbial contaminants. qPCR may be a focused-on approach that does not give a comprehensive viewpoint on the wide assortment of microscopic organisms, and quality contaminants display in biowaste, soil and wastewater streams [87]. Researchers consider both the focal points and impediments correlated with the 16S rRNA approach with that of the characteristic predisposition. There are outstanding distinctions between 16S rRNA screens and WMGS (whole metagenomic sequencing) strategies for organized and functional population profiling. For example, WMGS provides a thorough sample assessment by sequencing a large majority of random, small fragments in a shotgun approach individually, resulting in more sequencing coverage [63].

The quality ordered classification is rendered utilizing BLASTP look against the NCBI-NR database beneath a scale of e-value <10^−5^ for metagenome analysis. The repositories of KEGG (Kyoto Encyclopedia of Genes and Genomes) and COG (Clusters of Orthologous Groups) are utilized to bunch and classify the non-redundant quality set. Use of BLASTP look (Blast Version 2.2.28+) for COG and KEGG databases (e-value <10^−5^) is a valuable clarification of consistency. Based on a phylogenetic list of proteins expressed in various genomes of bacteria, archaea and eukaryotes, the COG database is commonly used for practical analysis on recent genomes and developmental study. By influencing the non-reductant content collection against the COG database, the percentage of usable categories of COG was established [62]. Examination of high-throughput sequencing information and a reasonable bioinformatics investigation approach in this manner played a really basic part within the examination of the microbial metagenome. These considered through bioinformatics tools such as MG-RAST, MetaVelvet, Genovo, etc., most of which borrowed from the areas of data mining, manufactured insights and measurements, have incredibly enhanced our information on microbial compositions and network-based relationship examinations [88]. Qi et al. [89] have utilized the metagenomics by utilizing the Illumina MiSeq high-throughput sequencing of the 16S rRNA quality to uncover the composition of the microbial community. Advance investigation of the shotgun metagenomic sequencing comes about uncovered a *Scedosporium* beginning CYP450 encoding quality, assigned cyp450q1 (GenBank no. MK388855), which offers 99% amino corrosive arrangement likeness (six amino corrosive changes among 525 amino acids) with that of the already detailed short-chain vaporous alkanes and ethers degradation-associated CYP450 quality CYP52L1 (Gen Bank no. AY438638) from Graphium ATCC 58400 [90].

RETRACTED

Employing a metagenomics approach the relationship between nitrogen expulsion execution and nitrogen change quality sort and abundance, as well as dispersion of important qualities in copious genomes are assessed. This allowed an appraisal of the ordered dispersion, plenitude and genotypes of the prevailing individuals of the community counting anaerobic alkali oxidation microscopic organisms and other individuals of the community [67]. Shotgun metagenomics arrangements are preprocessed for quality sifting of peruses and expulsion of a contaminant peruses (human and/or PhiX genome) utilizing Trimmomatic 0.36 and Bowtie2 (GRCh_38PhiX database) through the Knead Data wrapper program with ‘SLIDING WINDOW: 4:20, MINLEN 150’ parameters [67]. To perform metagenomics and metatranscriptomics, the primary step is to disconnect high-quality DNA and RNA from assorted tests. To date, there are two commonly utilized sequencing stages for metagenomics and metatranscriptomics: the Roche/454 stage (out of trade currently) and the Illumina framework (https://www.illumina.com). Some considers have moreover attempted the Pacific Biosciences (PacBio) stage and the Ion Torrent stage (https://www.thermofisher.com). For metagenomic and metatranscriptomic library development, Illumina gives a wide assortment of commercial packs. A few programs have been created for this step, primarily counting Trimmomatic, PRINSEQ, FASTX-Toolkit (http://hannonlab.cshl.edu/fastx_toolkit/), and NGS QC Toolkit. Among these programs, Trimmomatic may be an adaptable and proficient preprocessing apparatus that is particularly planned for Illumina yields and can create results prevalent to, or at slightest competitive with, other programs such as PRINSEQ and Fastx-Toolkit [71].

On the other hand, Motro et al. [88] developed the workflow of Microbial Metagenomics Deride Scenario-based Test Reenactment (M3S3) which permits clients to produce simulated tests from simple peruses. The M3S3 yield could be FASTQ or FASTA deride check. M3S3 is tested by creating virtual tests for 10 challenging irresistible illness scenarios, including a foundation framework with pathogens counting blends spiked in silicon. M3S3 is competent in creating on-demand simulated tests, reenacting a variety of complexity-changing symptomatic scenarios. The M3S3 instrument can subsequently bolster the improvement and approval of standardized metagenomics applications. Li et al. [91] have given a Bayesian system for genotype estimation for blends of numerous microscopic organisms, named as Genetic Polymorphisms Assignments (GPA). Recreation results appeared that GPA has diminished the wrong revelation rate and mean absolute error in CNV and single nucleotide variation (SNV) recognizable proof. This system was approved by whole-genome sequencing and Pool-seq information from *Klebsiella pneumoniae* with numerous microscopic organism’s blend models, and appeared the high precision within the allele division discoveries of CNVs and SNVs in AMR qualities between two populaces. The quantitative consider on the changes of AMR quality division between two tests appeared a great consistency with the AMR design watched within the person strains. Moreover, the system at the side of the genome explanation and populace comparison apparatuses have been coordinated into an application, which might give a total arrangement for AMR quality recognizable proof and measurement in un-cultural clinical tests.

RETRACTED

## 6. Quantifying the contribution of microbial immigration in ecosystem

Microbial populations in any environment be it natural or engineered play major roles in the biogeochemical cycles [92,93]. Different methods have been established, including the niche and neutral hypotheses, to investigate how different microorganisms aggregate into a population and add up to the ecosystem’s capacity [94]. Immigration is amongst the major stochastic processes in the neutral theory of biodiversity and biogeography, which together with death and birth alters population assemblage [95]. This is referred to as migration [96] and was originally used in macroecology to determine the rate of new species reaching a remote island from the closest landmass, i.e. the likelihood of colonization, which plays a critical role in maintaining the balance of faunal diversity of the island [97]. Since the definition of immigration can vary significantly [95], this review adopts the one previously used by Bell [98] and characterizes it as the procedure for introducing a microbial entity to a local community from the metacommunity species pool, which comprises of a lot of communities truly connected by immigration and which can exchange colonies of different species as well.

RETRACTED

One such commonly used, the equivalent word is dispersal [99–101]. While there may be some difference between dispersal and immigration in a particular context and one may even integrate the other [95], there is still no consensus on its differentiation. Throughout natural microbial processes, the shift from the upstream to a downstream network can be easily shown by the immigration of microbes from African dust to European marine condition [98], from flowing waters to woodland lakes [99] and also from river water to offshore environment and estuarines [100]. Immigration occurs more frequently in engineered conditions than in natural environments. Microorganisms found in various sources, such as surface and groundwater supplies, act as inocula in drinking water systems (Figure 6(a)) to propagate populations along the treatment procedure [99]. Microorganisms occurring on certain treatment systems, such as filters or reactor wall surfaces, can subsequently be released during or after processing [102] to the delivery units that depend on whether or not disinfection has occurred [103,104]. Bidirectional immigration amidst the water process and the biofilms on the inner pipe surface is feasible in the distribution network [105], which can further be elevated via stagnating the water [106]. Another case of microbial immigration can be seen in the wastewater treatment plant (WWTP) (Figure 6(b)), on the grounds that different bioreactors are directly linked to each other, and the biomass transfer is greater than that in the natural environment. In WWTPs, microbes in raw sewage system [106] and trickling filters [105–107] were recorded to have an effect on the populations of downstream-activated sludge. The activated sludge biomass [108] also serves as an immigration source for the downstream anaerobic digester [109–111]. The effluent [112] from the WWTP will influence the water supply network [113], thus raising the number of microbes and antibiotic-resistant genes associated with the human gut [114]. While microbial immigration is reported very often in engineered water systems, it remains very challenging to answer to what degree immigration contributes to the assemblage and operation of the downstream community. In this study, focus has been made on the procedure assessing microbial migration using survey methods that are now being used and also in establishing the drawbacks related to them. Immigration is a process that can have a strong impact on microbial communities in natural and engineered environments as well. In any case, it remains a challenge to quantitatively assess the commitment of this procedure to the microbial diversity and its proper functioning in the receiving ecosystems [115,116].

RETRACTED

Many approaches such as shared microbial species counting, microbial source monitoring, and commonly used neutral community modeling rely on an abundance profile to predict the degree of coverage between upstream and downstream networks [117,118]. Therefore, they cannot propose the contribution of immigrants to the role of the downstream communities because individual immigrants are not taken into account after reaching the receiving environment. This impediment can be solved by using a technique that combines a couple of mass balance with the sequencing of DNA, i.e. ecogenomics-based mass balance. This determines the net growth rate of individual microbial immigrants and splits the whole group into several communities that add to a community’s production and inactive ones that have almost zero functional benefit. Linking immigrant activities to their abundance also offer quantifying the contribution of an upstream community toward the downstream one. Considering that only active communities may improve the accuracy of categorizing the main ecological parameters which guide the execution of the procedure by using various techniques such as machine learning.

## 7. Conclusions and future prospects

Metagenomics is a dynamic approach to identify the microbial world and has provided signiﬁcant advancement between the research group and industrial application with regard to knowledge and importance of non-cultural microbes. Functional metagenomics is an important technique to identify the metabolites source from non-cultivable microorganisms. However, functional metagenomics is still facing many challenges that are yet to be solved because this technology is passing from development stages. Improvement of a metagenomic technology has already revealed to be beneficial. Even in its early years, it recommended that there can be important rewards if suitable advancement and further optimizations are conducted. The emergence of many metagenomic branches confirms the advancement in the techniques along with rapid and economic feasible sequencing assessment and will also acknowledge the amplification of a very encouraging research area in microbiology, genetic engineering, molecular science, pharmaceutical and food industries. This review article provides brief overview of the aptitude of developing metagenomics technology to produce novel industrial products obtained from uncultured microorganisms. Subsequently, the recovery of beneficial metabolites, upcoming challenges in another research area, is the advancement of a customer requirement and economic feasibility as well as the viable end product that can be further produced at industrial scale. In addition, it can also sustain its activity when scaled up and can be obtained puriﬁed and formulated appropriately into a final end product and keep its stability during preservation and transportation. A successful association of various metagenomics-based approaches is a requisite for identifying the complication of microbial communities, biological system and correlation with environmental factors in the last few years. In conclusion, the advancement of new ‘metagenomics’ technologies could be a competent tool to identify the microbial communities, contingent it is made more understandable, better informative, multipurpose, and economically feasible.

RETRACTED

**Figure 1.** General process of metagenomic workflow.

**Figure 2.** Systematic presentation of several environmental factors influencing soil microbial diversity.

**Figure 3.** Systematic presentation of metagenomics.

**Figure 4.** Schematic overview of the flow of resistant microbes (bacteria) and resistance genes in the food supply chain.

**Figure 5.** An overview of biotechnological tools for microbial community analysis.

**Figure 6.** Illustration of potential microbial immigration in (a) waterbodies and distribution system, and (b) wastewater treatment plants.
